This article has been retracted.

# Biologically Synthesized Copper Nanoparticles Show Considerable Degradation of Reactive Red 81 Dye: An Eco-Friendly Sustainable Approach

**DOI:** 10.1155/2022/7537955

**Published:** 2022-07-16

**Authors:** Muhammad Asim Rafique, Adil Jamal, Zainab Ali, Shumaila Kiran, Sarosh Iqbal, Sofia Nosheen, Zulqarnain Ansar, Md Belal Hossain

**Affiliations:** ^1^School of Economics and Management, Yanshan University, Qinhuangdao, Hebei Province, China; ^2^Sciences and Research, College of Nursing, Umm Al Qura University, Makkah-715, Saudi Arabia; ^3^Government Health Department Sialkot, Sialkot, Pakistan; ^4^Department of Applied Chemistry, Government College University, Faisalabad-38000, Pakistan; ^5^Department of Environmental Science, Lahore College for Women University, Lahore, Pakistan; ^6^Department of Plant Pathology, Faculty of Agriculture, Sher-e-Bangla Agricultural University, Sher-e-Bangla Nagar, Dhaka 1207, Bangladesh

## Abstract

*Diospyros kaki* leaf extract was used in this study as a favorable basis for the synthesis of copper nanoparticles (Cu NPs). X-ray diffraction (XRD) and UV-visible spectroscopy approaches were used to characterize the biologically synthesized copper nanoparticles. The XRD analysis showed that copper nanoparticles were face-centered cubic structure. Various experimental levels like conc. of dye, concentration of Cu NPs, pH, reaction time, and temperature were optimized to decolorize reactive red 81 dye using the synthesized Cu NPs. Reactive red 81 dye was decolorized maximum using Cu NPs of 0.005 mg/L. Additionally, reactive red 81 dye was decolorized at its maximum at pH = 6, temperature = 50°C. Our study reported that chemical oxidation demand (COD) and total organic carbon (TOC) deduction efficacies were 74.56% and 73.24%. Further degradation study of reactive red 81 dye was also carried out. Cu NPs have the ability and promising potential to decolorize and degrade reactive red 81 dye found in wastewater.

## 1. Introduction

Water is one of the most abundant natural resources on the planet, but just 1% of it is usable by humans [1, 2]. In the water supply system, continuing pollution of freshwater resources is a critical concern [3]. The textile sector makes a substantial contribution to the global economy and employs a huge number of people [4, 5]. Textile and garment sectors emit toxic waste high in organic compounds, especially colors, which are the principal outputs to the production process [6]. To discharge of dye-containing effluents, they have to go through a thorough preprocessing procedure that safeguards the human health and the environment [7–9]. Chemical, environmental, and toxicological aspects influence the numerous therapy options available. Adsorption [10], electrochemical [11], photodegradation [12], and bioremediation are some of the methods exploited in these investigations [13]. Wastewater treatment and drinkable water can assist to address these problems [14], but current treatment methods are unable to completely remove new contaminants and meet high water quality standards [15]. Moreover, current treatment technologies have serious flaws, such as a higher energy demand, poor pollutant removal, and harmful sludge development [14]. Biological wastewater treatment is widely utilized, although it is slow and can occasionally result in microbe toxicity as a result of toxic chemicals [16, 17].

Nanomaterials can be made in a variety of ways [18]. For the detoxification of industrial wastes, various effective, sustainable, and cost-effective nanomaterials with various features have been developed [19, 20]. Copper nanoparticles (Cu NPs) have been found to be effective in the breakdown of organic contaminants. Metallic nanoparticles were found to enhance dye degradation via reductive [21] or oxidative [22] mechanisms. Furthermore, the C-N link between the amine group and the core benzene ring of the molecule might break, resulting in primary amines as waste [22]. Hydroxyl radicals are produced in these environments, and they act in a Fenton-like reaction on the oxidative destruction of organic contaminants. Physical and chemical methods for producing nanoparticles are costly, require complex processes, and result in pollution as well as low productivity [23].

Scientists are working on developing biologically produced nanoparticles derived from plant extracts [24–28]. Plant-assisted nanoparticles can also be used to cure a range of diseases [29]. Persimmon, or *Diospyros kaki*, is a tropical, deciduous, pulpy/fibrous fruit from the Ebenaceae group. It is commonly cultivated in warm regions of the globe, mainly China, Korea, and other Asian countries. *D. kaki* exhibits a number of medicinal effects, such as powerful radical sequestration and antigen lethality in the seed [30], anti-inflammatory action in the leaves [31], anticarcinogenic, antihypertensive [32], and antidiabetic properties [33]. The goal of the current study was to develop low-cost, environmentally friendly methods for degrading reactive red 81 dye. *D. kaki* leaf extract was used to make stable Cu NPs in the first stage. Following the optimization of experimental variables, the second stage involved using these stable Cu NPs for decolorization of reactive red 81 dye.

## 2. Materials and Methods

### 2.1. Experimental Plan

All of analytical-grade chemicals and reagents applied in this research were acquired on the local market. The copper nanoparticles (Cu NPs) were synthesized utilizing *Diospyros kaki* leaf extract and were characterized using physical methods. After which they were employed to decolorize and degrade direct red dye.

### 2.2. Preparation of Extract and Cu NPs

Leaves of *D. kaki* were collected from the native marketplace and were washed thrice using distilled water to eradicate adhered dust particles. The washed samples were dried in shade. Dried mass of these samples was grinded to fine powder. Fine powder of green leaf extract (10 g) was mixed in 500 mL distilled water and heated to 70°C for 20 minutes. Then, solution was later filtered with funnel and Whatman filter paper. Filtered extracts were cooled at room temperature and labeled and kept at 10°C [34]. Copper sulphate (0.1 M) was mixed with 30 mL of leaf extract of *D. Kaki* and further diluted to 400 mL with distilled water. Solution was agitated at 90°C for 3 hrs. The change in color with the passage of time indicated that copper salt was being reduced to copper nanoparticles. The blend was centrifuged for 20-25 minutes, and the residue (Cu nanoparticles) was dried for 12 hours at 145-150°C.

### 2.3. Characterization of Copper Nanoparticles (UV-Vis Spectroscopy and XRD)

The qualitative biosynthesis of Cu NPs was investigated using UV-visible spectroscopy. An ultraviolet-visible (UV-Vis) spectrophotometer was used to validate Cu nanoparticle production. The peak absorbance of synthesized Cu NPs was measured in the spectrum region of 300-800 nm wavelengths. Shimadzu-Scientific Instruments (SSI), Kyoto, Japan, used the XRD 6000 series to obtain X-ray diffraction peaks utilizing a nickel filter and Cu-Ka target. The spectra were gathered in two ranges: 25-55 and 0-150 for strength indices. The average crystallite size of Cu NPs can also be measured utilizing the following equation of Debye-Scherrer:

*D* = *kλ*/*β* Cos *θ*.

*D* = average crystallite size (nm).

*k* = Scherrer constant with a value from 0.9 to 1.

*λ* = X − ray wavelength.

*β* = full width of half maximum.

*θ* = Bragg diffraction angle (degrees).

### 2.4. Experimental Procedure

100 mL of reactive red 81 dye solution (0.01%) was taken, its pH was attuned to 6.1 mg of copper nanoparticles that were added into it, and the reaction mixture was kept at 45°C for ninety minutes. The reaction′s progress was checked by taking little volume of reaction mixture after every 15 minutes and measuring its maximum absorbance (*λ*_max_) using a spectrophotometer [35]. Reactive red 81 dye level was changed from 0.01-0.05%, and copper nanoparticle dosage was altered from 0.001-0.01 g/L. pH level was adjusted from 4-8 and temperature from 40-70°C. All factors were elevated by the similar procedure by varying only one factor at a time.

### 2.5. Chemical Analysis

All experiments regarding decolorization were done in triplicate UV-visible spectroscopy was used to assess absorbance at 450 nm being measured. The following formula was used to calculate the efficacy of decolorization (%) for all parameters.

(1) $$\begin{array}{c} \text{Decolorization}\left(\%\right)=\frac{\left(I-F\right)}{I}\times 100, \end{array}$$

while *I* is the absorption at zero time, and F is the last absorption of the degraded color.

### 2.6. Mineralization Analysis and Degradation Study

Dye solution was evaluated using TOC and COD measurements. Vials were used to determine COD. These were filled with 3.6 mL of catalyst solution (silver sulphate in conc. H_2_SO_4_), a digesting solution of 1.5 mL (K_2_CR_2_O_7_ in acidified HgSO_4_), and 2.5 mL of reactive red 81 dye solution. In deionized water, a blank sample with all materials was also prepared instead of a reactive red 81 dye sample. The vials were placed at 150°C for 120 minutes. The vials were then cooled at room temperature, and the absorbance was recorded at 600 nm. A vial was filled with 1.6 mL concentrated H_2_SO_4_, 1 mL K_2_CR_2_O_7_ (2 N), and 4 mL reactive red 81 dye sample to determine the TOC value. The same sample was made with all ingredients except the dye solution, which functioned as a blank. The digestion vials were kept at 110°C for 90 minutes. The vials were then cooled at room temperature, and the absorbance at 590 nm was recorded [36]. For a precise measurement of the sample, the absorbance of the blank sample was subtracted from the absorbance of the sample.

COD and TOC values were estimated using the formula given below:

(2) $$\begin{array}{c} \frac{\text{TOC}}{\text{COD}}=\text{SF}\times A. \end{array}$$

When SF stands for standard factor, *A* stands for absorbance, and standard factor can be determined as follows:

(3) $$\begin{array}{c} \text{Standard factor}=\frac{\text{Conc}.\text{ of standard}}{\text{absorbance}}. \end{array}$$

The disintegration of reactive red 81 dye was measured in various phases involving the cracking of various connections and development of different moieties.

### 2.7. Statistical Analysis

All the parameters in experiments were performed in triplicates. Averages of triplicates were calculated. Results were computed using standard error and standard deviation mean.

## 3. Results and Discussions

### 3.1. Characterization of Copper Nanoparticles and Scanning of *λ*_max_

XRD was used to characterize the copper nanoparticles.  Figure 1 shows the XRD patterns for Cu NPs produced with *D. kaki* leaves extract. The graph shows powerful and strong peaks, indicating a crystalline face-centered cube (FCC) phase of produced Cu NPs. The strength of a solution can be determined by determining absorbed quantity. A UV-visible spectrophotometer was used to determine the wavelength of maximum absorption (*λ*_max_). The maximum wavelength was reported to be 450 nm (Figure 2).

### 3.2. Role of Experimental Conditions for Decolorization of Reactive Red 81 Dye Solution

Decolorization of reactive red 81 dye was involved the optimization of parameters like concentration of dye solution, concentration of Cu NPs, pH, and temperature.

#### 3.2.1. Effect of Concentration of Dye and Catalyst (Cu NPs) for Decolorization of Reactive Red 81 Dye Solution

Various amounts of reactive red 81 dye (0.01-0.05%) have been used in the ongoing study. Optimum decolorization (72.7%) of reactive red 81 dye was obtained at a dosage of 0.02%. Dye removal was reduced as the amount of reactive red 81 dye was increased (Figure 3). A greater number of dye molecules may self-associate, giving the medium a turbid appearance. Moreover, larger substrate concentrations may cause the catalyst to be inhibited, reducing the rate of the reaction [37–39]. Removal of dye was inhibited only when amount of reactive red 81 dye was high due to turbulence in the sample medium and the substrate acting as a blocker. The catalyst's efficiency is reduced when the amount of red 81 dye is at greatest [40–42].

In the current investigation, a variety of catalysts were being used. The % age of dye decolorized improved from 58.4 to 78.2% when catalyst level was raised from 0.001 to 0.005 g/L (Figures 3 and 4). As a consequence, it was found that the best acceptable catalyst dose for reactive red 81 dye decolorization is 0.005 g/L Cu NPs (Figure 4). The rate of dye decolorization increases as the catalyst concentration is increased. The dosage of Cu nanoparticles applied affects dye decolorization significantly [43]. The explanation for this is that as the concentration is raised, the number of active sites rises [44]. There will be no further development in rate of the reaction when the energetic sites of catalytic agents are entirely saturated with dye particles [45]. Increasing catalyst levels might cause turbulence in the solution due to a decrease in reaction rate [46].

#### 3.2.2. Effect of pH and Temperature for Decolorization of Reactive Red 81 Dye Solution

The dye solution's pH is important since it affects the dye's decolorization time and can modify the type of the charge density on the adsorbent's surface. In this work, we did a sequence of catalytic assays with pH levels from 4-8, whereas the other parameters stayed persistent. As the pH climbed from 4 to 6, the decolorization of the dye understudy increased from 57.9% to 86.1% (Figures 3 and 5). Rises in pH up to 8 caused a reduction in dye clearance over time (Figure 5). Increases in pH up to 8 resulted in a gradual decrease in dye removal (Figure 5). Fewer dye molecules are deposited on the catalytic surface because dye molecules are protonated at quite lower pH. At pH 6, attraction interactions between negative and positive charged catalytic surfaces interfaces were detected, indicating the highest interacting forces amongst dye nanoparticles at this pH [47, 48]. It is worth noting that the pH of the aquatic component has a significant impact on the adsorbent's charge [40]. In addition, catalysts have a pH value that is ideal for maximum catalytic potential [49]. Catalyst alteration can occur at pH levels greater than the optimum [50].

Experimental studies with an optimum dosage of Cu NPs (0.005 g/L) at temperatures ranging from 40-70°C have been performed out to evaluate the influence of temperature on the decolorization of reactive red 81 dye. As the temperature is increased from 40-50°C, the efficiency of dye decolorization rises from 76.3% to 87.8%, demonstrating that the catalytic action of Cu NPs is sensitive to temperature (Figures 3 and 6). The decolorization of the dye was reduced by up to 69.6% by raising the temperature to 70°C. As a consequence, 50°C was shown to be the best temperature for best dye removal of reactive red 81 dye by Cu nanoparticles (Figure 6). One theory is that catalysts have a large number of active regions for stimulating activities. Only at a certain temperature do catalysts achieve significant catalytic effect [40]. Temperatures that exceed the optimal value might cause permanent changes in the three–dimensional form of catalytic agents, resulting in declining the catalytic activity decline [51]. Our findings show that high temperature causes a decrease in dye decolorization (Figures 3 and 6). Temperature increases may cause a shift in the three-dimensional form of catalyst agents, reducing their dye adhesion ability [52].

#### 3.2.3. Mineralization Study

For the management of reactive red 81 dye utilizing Cu NPs as a catalyst, the mineralized efficiency was evaluated utilizing quality control metrics like COD and TOC. The COD and TOC of reactive red 81 dye solution were measured. % decrease in COD and TOC was calculated throughout a series of contact times from ten to seventy minutes. When the contact duration is amplified from 10-50 minutes, the %decrease of these metrics rises (Figure 7). COD and TOC levels decreased as the duration of contact was lengthened to 70 minutes (Figure 7). The products of a reaction might function as inhibitor, slowing down the speed of the process [53]. As indicated by higher COD and TOC removal values, Cu NPs not only decomposed but also mineralized our dye molecule and the other generated reaction intermediates formed at various stages of catalytic reaction [40, 54].

#### 3.2.4. Dye Degradation Study

Copper nanoparticles were employed to degrade direct red 81 dye which broke down the chromophore group firstly (Figure 8). The direct red dye's ring structure was later deteriorated. Intermediate products (carboxylic acids, aldehydes, and alkane) were generated once the dye molecule was degraded. During the mineralization, the basic substances such as carbon dioxide and water molecules were produced [24, 54].

## 4. Conclusion

Agro-waste stuff might be an excellent source of nanoparticles. Cu NPs were made physiologically using an aqueous extract of *Diospyros kaki* leaves. UV-visible and XRD analyses were used to characterize Cu NPs. Cu NPs were utilized to decolorize reactive red 81 dye. The dye decolorized up to 87.8% at 0.02% dye concentration, pH 6, and 0.005 g/L copper nanoparticle concentration at 50°C. COD and TOC levels were found to be 74.56% and 73.24%, correspondingly. The dye breakdown process produced the most basic components. Plant extracts could be employed in future investigations to produce additional metal oxide nanoparticles in a more environmentally friendly manner. So, it can be concluded that Cu NPs can potentially be employed to remove other notorious dyes present in industrial wastewater to eliminate their toxic effects, hence, saving the aquatic and terrestrial lives.

## Figures and Tables

**Figure 1:** Characterization of copper nanoparticles by XRD.

**Figure 2:** UV-vis spectroscopy result (*λ*_max_) of direct red 81 dye.

**Figure 3:** Decolorization of synthetic direct red 81 dye solution using Cu nanoparticles as a catalyst.

**Figure 4:** Decolorization of synthetic direct red 81 dye solution copper nanoparticle as catalyst.

**Figure 5:** Decolorization of synthetic direct red 81 dye solution at different pH using Cu nanoparticles as a catalyst.

**Figure 6:** Decolorization of synthetic direct red 81 dye solution at different temperature using Cu nanoparticles as a catalyst.

**Figure 7:** Effect of catalytic treatment interaction time on wastewater quality parameters.

**Figure 8:** Proposed degradation pathway of direct red 81 dye.

## Data Availability

All the data relevant to this study are mentioned in the manuscript. There is no any supplementary data.

## Abbreviations

Cu NPs: Copper nanoparticles
XRD: X-ray diffraction
COD: Chemical oxidation demand
TOC: Total organic carbon
K_2_CR_2_O_7_: Potassium dichromate
HgSO_4_: Mercuric sulphate
H_2_SO_4_: Sulphuric acid.
